The article "Role of Extrinsic Cues in the Formation of Quality Perceptions" was published in 2022. Journal: Front Psychol.

# Role of Extrinsic Cues in the Formation of Quality Perceptions

**DOI:** 10.3389/fpsyg.2022.913836

**Published:** 2022-07-25

**Authors:** Anam Javeed, Mohammed Aljuaid, Zoya Khan, Zahid Mahmood, Duaa Shahid

**Affiliations:** ^1^Department of Management Sciences, University of Wah, Wah Cantt, Pakistan; ^2^School of Business Management, University Utara Malaysia, Kedah, Malaysia; ^3^Department of Health Administration, College of Business Administration, King Saud University, Riyadh, Saudi Arabia; ^4^Department of Management Sciences, Peer Meher Ali Shah Arid Agriculture University, Rawalpindi, Pakistan; ^5^Department of Management, College of Business Administration, King Saud University, Riyadh, Saudi Arabia; ^6^Hult International Business School, Cambridge, MA, United States

**Keywords:** cues, signaling theory, perceived product quality, consumer market, perceptions

## Abstract

Examining the quality perceptions of consumers has often been recommended as an international research paradigm. This study is grounded in the Pakistani consumer market to evaluate the impact of food packaging cues on perceived product quality. The moderating effect of consumer knowledge was also taken into consideration in the study. A signaling theory was used in the study for its established predictive power in consumer behavior, marketing, and various fields of research. Based on the essence of the signaling theory, this study hypothesized that food packaging cues cast a positive impact on perceived product quality and consumer knowledge moderates these relationships. By using the sample of 504 consumers, data were gathered using the mall intercept method following a multi-stage sampling technique. The responses were analyzed using Statistical Package for Social sciences (SPSS) and Smart Partial Least Square (PLS). The findings of this study unveil that the extrinsic cues' brand name, price, nutritional labels, and precautionary labels were positively and significantly related to the perceived product quality. However, the country of origin cast no impact on the perceived product quality. Consumer knowledge reflected a moderation effect on the relationships between brand name and country of origin with the perceived product quality whereas it exerted no moderation impact on the relationships of price, nutritional labels, and precautionary labels with the perceived product quality. As the results exhibit that Pakistani consumers rely on food packaging cues for perceiving a product, hence it is recommended that marketers and policymakers develop appropriate marketing strategies focused on the significance of food packaging cues.

## Introduction

The modern-day concept of consumer behavior revolves around the consumer who is the ultimate authority (Pearce, 2016; Chonpracha et al., 2020). This viewpoint makes it important for enterprises to gather a deeper comprehension of consumer perceptions for product differentiation in order to gain a competitive edge (Ravikanth and Rao, 2016). The product attributes provide an opportunity for the firms to develop their products as per the needs of consumers and develop product differentiation (Charlebois et al., 2016). Advertising cues impact the consumer attitude toward the product quality (Dawar and Parker, 1994). Packaging plays a pivotal role in marketing and a role of a silent salesperson to attract customers (Wang, 2013). The cues extended toward the consumer are of vital importance (Kim, 2008). The cues presented on the food packaging create an impact on the perceptions of the consumers and even small numerical differences presented on the package can positively affect the quality perception (Spence and Velasco, 2018). Cues that attract the consumer can trigger the competitiveness among the products and brands (Bauer et al., 2012; Mugge and Schoormans, 2012). Dissimilar to conventional advertising in which consumers come across the promotional messages at various places, the buyers notice the packaging of the product usually at the sale points and trade stores (Wigley and Rachel Chiang, 2009). Especially with fast-moving consumer goods, consumers rely on the food packaging cues when picking a product (Honea and Horsky, 2012).

The article "Role of Extrinsic Cues in the Formation of Quality Perceptions" was published in 2022. Journal: Front Psychol.

In the case of packaged foods, consumers are more cognizant due to frequent consumption as food has a direct impact on the health of the person. The food manufacturing companies that introduce packaged food items embed the favorable cues in the packaging (Magnier et al., 2016). The processed packaged foods in Pakistan are becoming popular due to the increasing income and modernization of living (Ayyaz et al., 2011). The increasing drift of urbanization in Pakistan is giving a boost to the packaged food industry. Urban consumers are more inclined toward the use of packaged food items. The quality of packaged food is under debate in the food industry, public, as well as among researchers (Moslehpour and Huyen, 2014). Food quality has become a topic of interest because of the following reasons. First, the scarcity of food has engaged the attention of the researchers to probe into the quality issues (Moslehpour and Huyen, 2014). Second, the general public has become more concerned about the quality of food (Ergin et al., 2014). In recent times, the environment has emerged as a hot issue for societies and governments, in addition to business organizations. Its significance originates from escalating environmental degradation such as solid wastes, ozone depletion, global warming, and air pollution. It is observed that different activities of business organizations such as sourcing, manufacturing, logistics, and marketing have a negative impact on the environment and are also considered to be the source of most the environmental problems (ElTayeb et al., 2010). Because of the nature of their products and the markets in which they compete, managers always perceive their company as being unique; thus, they consider their problems as being different to those faced by other companies. However, experience shows that the underlying problems faced by most companies are essentially similar, namely the need to meet delivery dates, ensure product quality, reduce costs, enhance the product specification, etc. What is unique to a specific company is the particular combination and magnitude of these problems. Therefore, if two companies of a similar size and structure are competing in the same market, one may find that delivery performance is its major problem, whereas the other may consider that product cost is its biggest worry.

The article "Role of Extrinsic Cues in the Formation of Quality Perceptions" was published in 2022. Journal: Front Psychol.

### Problem Identification and Research Questions

Quality perception of buyers has been a major topic of interest in previous literature (Rahman et al., 2017). The previous attempts are relatively fragmented and do not consider a comprehensive set of packaging cues to describe the quality perceptions of the buyer (Lähteenmäki et al., 2010; Kelley et al., 2015). It has been argued that even though buyer intends to perform a certain behavior but there is a possibility that they might not be able to purchase without necessary informational cues (Ajzen, 1991). The buyer characteristics can vary from one market to another market due to cultural alterations. Cultural factors play a pivotal role in buying choices. By exploring the variables and their nexuses with the theories, the Pakistani cultural context can yield worthwhile results. Thus, the major problem that this study aims to address is how the extrinsic product cues of precautionary label, country of origin, brand name, and price impact the perceived product quality.

As the life trends are changing in Pakistan, the needs and wants are changing accordingly. The phenomenon of modernization is taking place due to a heightened level of awareness and globalization (Qadeer, 2006). The level of education and awareness is making the Pakistani buyers acquainted with the food packaging, labeling, and the information being presented on it. Even though the Pakistani buyer is becoming aware of labels, some of the labels are new to Pakistani buyers, for instance, nutritional labels and precautionary labels (Sohail, 2005). The knowledge of the Pakistani consumers about the food packaging labels is relatively low when compared with the developed country buyers but progressively increasing.

The article "Role of Extrinsic Cues in the Formation of Quality Perceptions" was published in 2022. Journal: Front Psychol.

Taking into consideration the present scenario of Pakistani buyers regarding the packaging cues, a model has been established to study the impact of brand name, price, and country of origin on the perceived product quality. Consumer knowledge is employed as a moderator in order to find out how the progressively increasing level of knowledge impacts the formation of perceptions regarding product quality and food packaging cues.

Therefore, this study focuses on answering the following two main research questions:

i. How does the extrinsic cues impact the perceived product quality?
ii. Does the consumer knowledge moderate the relationship between extrinsic cues and product quality perception?

## Literature Review

In this section, relevant literature has been discussed, and hypotheses have been developed accordingly. The nexus of perceived product quality with brand name, country of origin, price, and precautionary label have been discussed in the following subsections. The impact of consumer knowledge as a moderating variable has also been discussed in this section.

### Brand Name

A brand name is quite effective in creating product quality perceptions (Javeed et al., 2017). A well-established brand name can be helpful in the formation of purchase intention of buyers toward the products (Rungtrakulchai, 2018). The brand name possesses the potential to cast a positive impact on the perceptions of the customers. The positive perception of buyers for the product can in turn lead to the formation of purchase intention. Purchase intention refers to the tendency of a shopper to buy the brand (Diallo and Seck, 2018). It is also a key element for the long-term success of relationships (Sharma and Garg, 2016). With a well-established brand name, buyers generally have to spend very less time perceiving the quality of the product (Randhawa et al., 2017). The stout relationship between brand name and product quality perceptions motivates frequent buying behavior (Mishra et al., 2017). It has further been argued by Lewis et al. (2016) that the relationship between the brand name and the product quality perception is vital as a well complex issue and should be probed closely in various markets. The worth of the brand name in casting an impact on the preference formation and quality evaluations of the food has been stressed upon by Chovanová et al. (2015). The importance of the brand name as an important packaging cue and quality determinant has been stressed upon by Babcanová et al. (2012). It has been argued that the brand name influences not only the quality perceptions but also brand purchase (Ismail et al., 2012). Consuming branded food items provides the user with a sense of prestige (Zhou et al., 2020). A significant role of the brand name in the willingness to pay higher for a certain product has been argued by Holt (2002). A cross-country examination conducted by Zeb et al. (2011) between the brand name and the purchase intention yielded mixed responses among different countries where variables depicted positive, negative, and no relationship. Another study reported a direct significant nexus between the brand name and the social acceptance (Grewal et al., 2011). Moving on further, it has been observed that buyers in developing countries are far less brand conscious, and they prefer the cue of price over brand name (Shehzad et al., 2014). More recently, it has been reported that consumer evaluates the product of a reliable brand positively (Mascarello et al., 2015; Choi and Lee, 2019).

The article "Role of Extrinsic Cues in the Formation of Quality Perceptions" was published in 2022. Journal: Front Psychol.

Connelly et al. (2011) state that the signaling theory practically aids in the mapping of consumer behavior. The prior studies using the signaling theory considered consumer purchase behavior and the formation of quality perceptions through packaging elements serving as quality signals (Kirmani and Rao, 2000). According to the argument of Connelly et al. (2011), the signals extended toward the consumers are in the form of favorable cues regarding the product about to be sold. Furthermore, specifically in the arena of packaged food, the cues and attributes on packages tend to impact the perceptions regarding inexperienced quality. The cues present on food packaging in most recent times has played a major role in perceiving the quality (Fernqvist and Ekelund, 2014). According to the results produced by Loken et al. (2010b), brand name as an extrinsic cue casts a significant positive impact on the product quality perception. It is further confirmed that understanding the impact of brand name awareness assures the disclosure of proper information on the individual's quality perceptions (Babcanová et al., 2012). In another investigation, it is revealed that perceptions are influenced significantly by the food labels on packaging (Chovanová et al., 2015). There are numerous studies that have found a significant relationship between brand name and product quality perception (Loken et al., 2010a; Wei et al., 2020). The cue of the brand name can offer various different types of connections and meanings to the consumers in a manner that become a part of the consumer's knowledge (Bao et al., 2008). In order to establish connections and attachments, marketers tend to spend a considerable amount of resources to instill favorable associations (Yan et al., 2012). The rising environmental concerns within the global consumers have also heightened the demand for high quality products. The growing environmental concerns among consumers around the globe have spurred the demand for greener products (Schmuck et al., 2018).

The article "Role of Extrinsic Cues in the Formation of Quality Perceptions" was published in 2022. Journal: Front Psychol.

**H**_**1**_**:** Brand name has a significantly positive impact on the perceived product quality.

### Country of Origin

Internationally, the origin of the product labeling impacts the perceptions of the consumers of every age group (Velčovská and Hadro, 2018). It has been shown that the country of origin effect varies with the consumers belonging to different countries (Insch and McBride, 2004). Looking into the context of Pakistan, the country of origin has a positive association with product quality judgments and buying decisions (Khan and Bamber, 2008). The literature on the Pakistani consumers regarding the impact of country of origin on quality perception is less when compared with the data regarding the variable in the rest of the world (Ghani et al., 2007; Saeed et al., 2013; Saeed and Aslam, 2015; Murtaza, 2016). Investigating the extent of the relationship of the country of origin with the product quality perception along with other product packaging cues would be an important theoretical contribution to literature due to the scarcity of literature (Hien et al., 2020). The image of the country of origin is associated with the product that develops the perceptions of the consumers (Mørkbak et al., 2010). The country of origin logo signals the general perceptions and imagery which the consumers form about the quality of the product (Türkekul et al., 2010). The signaling power of the country of origin cue influences the consumer's evaluation of the quality of the enclosed product which has further been emphasized by Thøgersen et al. (2017). The country of origin is the effect of the product, which describes the extent to which the consumer's product evaluations are signaled by the country of origin logo (Lee et al., 2013). The country of origin of the product has a direct impact relationship with the perceived quality by signaling the quality (Diamantopoulos and Zeugner-Roth, 2010). There exists a direct influence of country of origin on the perceived quality and purchase intentions (Rezvani et al., 2012). It has been observed that country of origin has a varied level of influence on the quality perceptions of the consumers (Pappu et al., 2005). The prior studies have verified the relationship between the country of origin label and the product quality perceptions (Kalicharan, 2014). On similar grounds, the affiliation has reported significant results in various other studies conducted by Andéhn and L'Espoir Decosta (2016). Various other studies have exhibited that country of origin labels cast a positive impact on the perceptions of quality in the minds of the consumers (Rezvani et al., 2012). Provided the given variety of food products and the overflow of information in the market, certification labels are intended to encourage consumers to select healthier and more sustainable product options. Although there is a number of other labels, the country of origin label is considered to be mandatory (Li et al., 2017).

The article "Role of Extrinsic Cues in the Formation of Quality Perceptions" was published in 2022. Journal: Front Psychol.

Taking into consideration of the previous studies that have proved the positive effect of country of origin on the perceived product quality like Rezvani et al. (2012) and Kalicharan (2014), this study hypothesizes that:

**H**_**2**_**:** Country of origin label has a significantly positive impact on perceived product quality.

### Price

The cue of price has been tested in the past; however, the outcomes are mixed and varied, therefore inconclusive. For instance, Kim et al. (2009) reported a significant relationship; however, Parguel et al. (2016) reported that price does not always cast an impact on quality perceptions. Price is a salient cue of the product whose importance cannot be denied as it serves as a quality cue and the buyer perceives the eminence of the product from the price (Bolton et al., 2010). It has been reported in past investigations that consumers have a prevailing belief of the fact that higher quality products are worthy of high prices whereas the less expensive products are lesser in quality (Grunert et al., 2004). Conversely, in other studies, price is found to be overridden by other informational cues such as brand name and packaging information (Homburg et al., 2005). The influence of the price as a quality indicator is much more powerful when a consumer has less knowledge (Weisstein et al., 2013). The consumer perceives the quality of product by the signals that the price cue display (Riley et al., 2004). In another study, the perceived quality of the product is signaled by price cues along (Truong et al., 2009). Contrasting evidence has been presented in another study in which it is mentioned that the consumers perceive that they are offered value against the higher price they pay for the product (Fassnacht et al., 2012). The brands should keep an optimal price to signal for best quality of the product (Kapferer, 2012). Luxury brands can signal luxurious effects of the product by using a higher margin of product (Kapferer, 2012). The price level is an empirical variable that can be used to signal the perceptions and attitudes of the consumer toward the product (Riley et al., 2004).

The article "Role of Extrinsic Cues in the Formation of Quality Perceptions" was published in 2022. Journal: Front Psychol.

Studies have shown that consumers utilize price as a major quality indicating cue in a purchasing situation (Kostyra et al., 2016). Another investigation proved that price has a significant impact on the perceived product quality (Flach, 2016). Numerous studies have confirmed the relationship that the price tag is a strong cue for quality judgment of the product prior to the usage (Mathe-Soulek et al., 2016). Another study has proved that price has a strong impact on product quality perceptions (Ghasemi et al., 2016). The cue of price has been recognized to play a substantial role in the formation of product quality perceptions. Moving on further, it has alo been confirmed that price has a positive influence on the perceived product quality (Parguel et al., 2016). A significant nexus between price and product quality perception has been reported by Zeithaml (1988). The price is an indicator of quality and instills a sense of prestige (Weisstein et al., 2013). There is a significant relationship between price and brand image (Kluge and Fassnacht, 2014). It is asserted that price display impacts quality perceptions (Doss and Robinson, 2013). In the previous years, the environmental concerns are being addressed by the companies, and consumers seem to pay a little more for the environmentally friendly products. The managers and policymakers should not only have economic concerns but also consider social and environmental issues while determining the price of the product.

Therefore, the third hypothesis for this study can be inferred as:

**H**_**3**_**:** Price has a significantly positive impact on perceived product quality.

### Precautionary Label

Precautionary labels are basically the health warnings that address the hypersensitivity issues of the consumers (Chiuve et al., 2011; Hancock et al., 2020). However, the precautionary labels are not only a source of information to the consumer but also a marketing edge for the companies that display them (Turnbull et al., 2015). Based on the argument of the aforesaid scholar, it can be derived that the consumers consider the precautionary labels for making the perceptions of quality regarding the packaged food. The finding on this relationship is mixed. Few studies find a negative relationship between the precautionary label and the quality of food (De Blok et al., 2007). On the other hand, few studies have found a positive relationship between precautionary labels and the quality of food (Fox et al., 2009). As other extrinsic cues discussed in the study namely brand name, country of origin logo, and price, precautionary labeling also tends to signal the quality of the product hence complying with the basic assumptions of signaling theory. There are many studies pertaining to food labeling which bring ideas for the manufacturing industries of food products in the aspect of labeling (Abdul Latiff et al., 2013). According to the survey, the consumers have less understanding of label reading and mostly the people with severe allergic reactions such as asthma and unconsciousness tend to read the precautionary label more (Cochrane and Ebmeier, 2013).

The article "Role of Extrinsic Cues in the Formation of Quality Perceptions" was published in 2022. Journal: Front Psychol.

Therefore, this study hypothesizes that:

**H**_**4**_**:** Precautionary labels cast a significant impact on perceived product quality.

### Consumer Knowledge

The strength of the independent and dependent variables can be altered by a third variable known as a moderator (Baron and Kenny, 1986). The moderator has the potential to enhance or reduce the forte of nexus between independent and dependent variables. It can even change the relationship between the two constructs in both positive and negative ways (Lindley and Walker, 1993). Consumers give particular importance to nutritional facts but the information on the labels may not always communicate the intended message (Wills et al., 2009; Ahmad and Guzmán, 2020). Although the theoretical linkage among the extrinsic cues, perceived product quality, and moderating role of consumer knowledge is comprehendible (Alba and Hutchinson, 2000; Veale, 2008), not many studies have employed consumer knowledge as a moderator. To test the moderating effect of consumer knowledge on the entire image variables one by one, the following are the hypotheses to be tested:

**H**_**5**_**:** Consumer knowledge moderates the relationship between the brand name and the perceived product quality.

Previous studies by various researchers develop a consensus that the country of origin is a vital quality indicating cue. The long-term working memory presented by Ericsson and Kintsch (1995) says that the consumer integrates the new information with existing linkages in the memory. This integration of information results in the formation of long-term memory networks (Chiesi et al., 1979; Ericsson and Kintsch, 1995). The impact of consumer knowledge on perceptual processes has been studied by several researchers for instance (Jacoby et al., 1974; Charness et al., 2001). Hidalgo-Baz et al. (2017) argue that consumer knowledge impacts the perceptions of the consumers regarding the product; however, regional differences exist because the nature of the market differs all over the globe. Due to the increasing level of education in Pakistan, the consumer is becoming knowledgeable, and they are more likely to promote more healthful diets because more highly educated people access and process nutrition information more effectively (Latif et al., 2016). To understand the role of consumer knowledge as a moderator between the country of origin and the perceived product quality, it is hypothesized that:

**H**_**6**_**:** Consumer knowledge acts as a moderator between country of origin and perceived product quality.

The article "Role of Extrinsic Cues in the Formation of Quality Perceptions" was published in 2022. Journal: Front Psychol.

The knowledge possessed by the buyers regarding the product affects their perceptions (Yen et al., 2008). Taking into consideration the Pakistani context, the buyers are becoming more knowledgeable about their consumption choices (Latif et al., 2016). Although the knowledge level of the Pakistani consumers is increasing, the literature has very minimal support in this regard. Investigating the relation of consumers' knowledge as a moderator could yield some interesting insights regarding Pakistani consumers (Chuang et al., 2009). In a purchase situation, the ability of interpretation and accurate evaluation of the consumers about extrinsic and intrinsic cues may vary (Kardes et al., 2001). In a variety of situations, price is an attribute that the buyers use widely to evaluate the quality of the product (Kardes et al., 2001; Wansink, 2004). In order to analyze the moderating effect of the consumer knowledge in the relationship between price and perceived product quality, it is hypothesized in this study that:

**H**_**7**_**:** Consumer knowledge moderates the relationship between price and perceived product quality.

This integration of information results in the formation of long-term memory networks (Chiesi et al., 1979). The impact of consumer knowledge on perceptual processes has been studied by several researchers (Charness et al., 2001), and based on these studies, consumer knowledge casts an impact on the usage of extrinsic cues. Riley et al. (2013) argued that the price of the product is a multi-dimensional construct. In the study of Truong et al. (2009), the perceived higher quality of the product was reported to be an important and significant dimension among the other cues of brand name and store name. Contrasting evidence has been presented by Kluge and Fassnacht (2014) in which it is mentioned that the consumers perceive that they are offered value against the higher price they pay for the product. The usage of the precautionary label as a quality cue by the consumers has been confirmed by Voordouw et al. (2011). The precautionary labels are comprehensive and communicate uniform and explicit information which communicates the presence of any potential allergen (Voordouw et al., 2011). A major factor regarding precautionary labels and health claims is that consumers associate health-related perceptions with them (Fulgoni et al., 2009). As the literature suggests, the moderating role of consumer knowledge is rare in analyzing the relation between the precautionary label and the product perceived quality. Therefore, it is hypothesized that:

**H**_**8**_**:** Consumer knowledge acts as a moderator between precautionary label and perceived product quality.

The article "Role of Extrinsic Cues in the Formation of Quality Perceptions" was published in 2022. Journal: Front Psychol.

### Product Quality Perception

Product quality perception is a topic of interest in modern times (Priilaid et al., 2017; Gao et al., 2020). The concept of product perceived quality has been defined as “product perceived quality as a unique kind of association created in the mind of consumers which not only impact the brand associations on the minds of consumers but also the profitability of the manufacturer” (Aaker and Joachimsthaler, 2000). It has been emphasized that the perceived quality is dissimilar to the actual quality and comprises a higher-level abstraction (Zeithaml, 1988). The determination of consumer perceived quality leads to satisfied consumers (Chaudhary, 2014). The overall meaning of the perceived quality common in all the definitions is that “perceived product quality is the abstraction of the overall components of the product's both tangible and intangible” (Nath Sanyal and Datta, 2011). The quality traits can be defined as the tangible and intangible characteristics of the merchandise, which show an impact on the perceived product quality of the consumers (Kupiec and Revell, 2001). Extrinsic cues provide an imprint that resultantly forms the product perceptions (Dawar and Parker, 1994). For comprehending the expectations of the consumers regarding the quality, the product manufacturers need to absorb information related to the perceptions and assessments of the consumers (Main, 1994). Systematic research is needed to understand and comprehend the perceptions of consumers as it is not an easy chore (Ergin and Akbay, 2014). The use of extrinsic cues for instance brand name and price in various product categories has been confirmed by Moslehpour and Huyen (2014).

### Underpinning Theory: Signaling Theory

Within the literature on marketing, the extrinsic cues are taken as the indicators of quality for the enclosed product. The signaling theory was proposed by Spence (1973). Spence (1973) explained the concept of the signaling theory initially from the perspective of economics. The signaling theory was applied by Renwick et al. (2013) in the context of job suitability of the candidates. In recent days, the phenomenon of signaling has been extended to quality perceptions in the field of marketing. Various scholars have stated the importance of the signaling theory in the formation of mental mapping (Connelly et al., 2011). In a previous study, Kirmani and Rao (2000) stated that the signaling theory is worthwhile in reviewing the purchase behavior of the consumers and the formation of quality perceptions for the packaged products. The quality signals that are aimed toward the consumers and buyers are in the form of a cue regarding the product (Connelly et al., 2011). The main attention of the signaling theory is the lessening of information asymmetry between the sellers and buyers (Spence and Piqueras-Fiszman, 2012). The signaling theory can be referred to as the framework for understanding the buyers' viewpoint when exposed to the various types of quality signals (Fletcher-Brown et al., 2018).

The article "Role of Extrinsic Cues in the Formation of Quality Perceptions" was published in 2022. Journal: Front Psychol.

### Rational Choice Theory

The “Rational Choice Theory” elaborates that the important decisions of humans are taken in a way that benefits them the most. All the options are carefully screened by the consumers, and after that, they go on with their purchase. This is the premise of rational choice theory, which is widely discussed in economics and marketing and states that people tend to make decisions that maximize benefits while minimizing risks. The theoretical framework shown in Figure 1 depicts that the extrinsic cues can help to formulate positive perceptions regarding the product. The rational choices are generally made by the consumer on the basis of knowledge they possess regarding product.

**Figure 1:** Theoretical framework.

## Methodology

The research methodology used in the study has been described in the following sections.

### Population and Sample of Study

Sampling is a way to overcome the hurdles of collecting data from all of the population which is almost impossible in terms of time and money (Forza, 2010). The sample is selected on the basis of their characteristics and properties in order to generalize the outcomes (Uma and Roger, 2003). While conducting the investigations, it is practically impossible to collect data from a large population; hence, the sample is chosen. It has been argued that using an appropriate number of respondents as a sample for the study may save time and other resources (Uma and Roger, 2003).

Islamabad and Rawalpindi were selected as samples because they are major big cities of Pakistan having a dense and diverse number of people as inhabitants from all over the country, hence making the study generalizable. The combined population of Rawalpindi and Islamabad is approximately 4.4 million inhabitants. The sample has been bifurcated among the cities proportionately as listed in Table 1.

The article "Role of Extrinsic Cues in the Formation of Quality Perceptions" was published in 2022. Journal: Front Psychol.

**Table 1:** City wise sample size.

**City**	**Calculation**	**Proportionate sample size**
Islamabad	1,430,000/4,430,000* 504	163
Rawalpindi	3,000,000/4,430,000* 504	341

### Data Collection Procedure

The data collection for this study was carried out for several weeks after pilot testing. A self-administered questionnaire was used to collect the data from the Pakistani consumer market. In this study, the population of interest was general consumers visiting the shopping mall. To minimize the bias and to address the time issues as the number of visitors varies considerably across the day, the data collection time was split into two halves of the day (Sudman, 1980). Table 2 lists the proportionate sampling time- and day-wise.

**Table 2:** Proportionate sample time and day wise.

**Shopping center/city**	**Proportionate sample size on weekdays**		**Proportionate sample size on weekends**	
	**9 a.m−3 p.m**	**3 p.m−9 p.m**	**9 a.m−3 p.m**	**3 p.m−9 p.m**
C M/Isb	10	12	12	19
B C/Isb	3	9	16	22
K M/Isb	6	16	13	25
CSD Mall/Rwp	12	22	19	28
CSD Super Mall/Rwp	6	16	19	31
G V P Hyper mart/Rwp	9	22	25	32
R M/Rwp	13	16	34	37

### Survey Instrument

The variables used in this study have been adapted from the previous literature depending on the value of Cronbach's alpha. In addition to the advantage of higher reliability values, the adapted questions conveyed the exact meanings as the research was envisioned. The adapted scale was designed in a manner that would produce the exact desired responses. This adoption would reduce the time burden on the researcher in proportion to the analytical requirements of the survey (Biemer and Lyberg, 2003). This study used the Likert scale to measure the responses since this scale is widely used in various areas such as marketing and behavioral sciences. Employing the five-point Likert scale is as good as any other (De Winter and Dodou, 2010). The questionnaire has been constructed based on dimensions extracted from the literature. Table 3 lists the dimensions of the constructs and their sources.

**Table 3:** Dimensions of the constructs.

**Constructs**	**Dimensions**	**References**
Brand name	• Consistent quality • Social approval • Prestige	Jamal and Sharifuddin, 2015; Gracia and de-Magistris, 2016
Country of origin	• Sophistication • Superior quality	Qasem et al., 2016
Price	• Higher quality • Value for money	Wang, 2013
Precautionary label	• Awareness • Healthfulness	Ambali and Bakar, 2013
Consumer knowledge	• Objective knowledge • Subjective knowledge	Alba and Hutchinson, 2000
Perceived product quality	• Perceived healthfulness • Perceived safety and security • Perceived superiority	Asshidin et al., 2016

The article "Role of Extrinsic Cues in the Formation of Quality Perceptions" was published in 2022. Journal: Front Psychol.

### Common Method Variance

It is stated by Podsakoff et al. (2003) that common method variance is attributable to the method of measurement. In order to check the common method variance, Harman's single factor test has been applied in the study. If a considerable volume of variance exists then either one single factor might emerge or one factor might account for the covariance present among independent and dependent variables (Harman, 1976). The analysis shown in Table 4 clearly depicts that no single value accounted majorly for the covariance (the first factor explained 25.542%) which is clearly < 50%. The values suggest that the common method bias is not the main apprehension, and it is unlikely to inflate any relationships (Table 5).

**Table 4:** Total variance explained.

	**Component**	**Initial Eigen values**			**Extraction sums of squared loadings**		
		**Total**	**% of Variance**	**Cumulative %**	**Total**	**% of Variance**	**Cumulative %**
Raw	1	17.463	25.542	25.542	17.463	25.542	25.542
	2	5.687	8.318	33.860			
	3	3.009	4.402	38.261			
	4	2.811	4.111	42.373			
	5	2.530	3.700	46.073			
	6	2.444	3.575	49.648			
	7	2.059	3.012	52.660			
	8	1.646	2.408	55.068			
	9	1.589	2.325	57.392			
	10	1.420	2.077	59.469			
	11	1.293	1.891	61.361			

**Table 5:** AVE and composite reliability.

**Variables**	**Composite reliability**	**Cronbach's alpha**	**AVE**
Brand name	0.861	0.806	0.508
Country of origin	0.867	0.794	0.623
Price	0.861	0.800	0.553
Precautionary label	0.876	0.835	0.503

Composite reliability is the extent to which the items seek to designate the latent construct (Hair et al., 2010). The ideal value for composite reliability is suggested by Fornell and Larcker (1981) and Hair et al. (2010) is 0.70.

Another assessment to be considered in structural model evaluation involves the effect size (*f*^2^) of each relationship in the structure model, which allows researchers to evaluate the exogenous latent variable's incremental explanation of an endogenous latent variable. The effect size can be determined by calculating Cohen's *f*^2^ (Chin and Dibbern, 2010; Cohen, 2013). Table 6 lists the effect size of the variables.

**Table 6:** Effect size.

**Brand name (BN)**	**0.022**
**Country of origin**	**0.001**
**Price (PR)**	**0.008**
**Precautionary label (PL)**	**0.071**
**Consumer knowledge (CK)**	**0.010**

## Analysis

In order to analyze the data collected through questionnaires, SMART-PLS has been applied. The software has been used due to wide usage in social sciences study.

MacCallum and Austin (2000) described the details of different usage of SEM in psychological research. It is also applied in the sub-areas of social sciences like sociology (Yan et al., 2016), economics (Bansal et al., 2014), and marketing (Sheeraz et al., 2012; Li et al., 2017; Schmuck et al., 2018). It is equally applicable in observational and experimental research. There has been a critical issue about the generalizability of results in the community within the context of social sciences. It is also a sensitive issue about the appropriate selection of analysis techniques in a SEM. The main aim and mean to an end is the data analysis. The mean of data analysis is always subject to the nature of different relationships among different variables and also depend upon the researcher. There may be many means related to data analysis. This is really a critical matter about the mean that should be highly proper, useful, and highly supportive to obtain reliable results and to convince the readers about results.

The article "Role of Extrinsic Cues in the Formation of Quality Perceptions" was published in 2022. Journal: Front Psychol.

Previous studies that have worked with similar kinds of cues have for instance (Acebron and Dopico, 2000; Teas and Agarwal, 2000) worked with experimental design. This study has considered a quantitative research design for investigating the impact of extrinsic cues on product quality perception.

The basic information regarding the cities of Pakistan is shown in the table below.

### Reliability

Measuring the internal consistency of the items ascertained for the construct is termed reliability (Hair et al., 2011). Cronbach's alpha coefficient primarily tends to reflect the items' consistency and as such, higher Cronbach's alpha values indicate higher consistencies which further reflect a higher tendency to measure the intended construct (Khan et al., 2019; Awan et al., 2020). Convergent validity illustrates the homogeneity of the scale whereas discriminant validity refers to the heterogeneity of the constructs, that is, the extent to which the measure is unique from other measures (Malhotra and Galletta, 1999). Table 7 lists reliability test values.

**Table 7:** Reliability test.

**Serial no**	**Construct**	**Composite reliability**	**Cronbach's alpha**	**No. of items**	**Items**
1.	Brand name	0.861	0.836	5	BN1 BN2 BN3 BN4 BN5
2.	Country of origin	0.867	0.806	4	COO1 COO2 COO3 COO4
3.	Price	0.861	0.801	5	PR1 PR2 PR3 PR4 PR5
4.	Precautionary label	0.876	0.849	5	PL1 PL2 PL3 PL4 PL5
5.	Perceived quality	0.907	0.851	5	PQ1 PQ2 PQ3 PQ4 PQ5
6.	Consumer knowledge	0.920	0.916	5	CK1 CK2 CK3 CK4 CK5

### Validity Test

Even though the instrument possesses reliability but they do not necessarily imply the goodness of the measurements (Uma and Roger, 2003). The instrument might lack the aspect of validity. The two basic measures of validity are content validity and construct validity. The judgmental assessment regarding the questionnaire and its constructs by the experts is called the content validity. Construct validity is performed to ascertain that a test is evaluating the construct it was actually supposed to (Brown, 1983). To ensure the overall validity, construct validity is deemed necessary. Factor analysis was performed to ensure the construct validity (Muthén and Kaplan, 1985; Mulaik, 2009). Sampling adequacy was measured by using the KMO (Kaiser-Mayer-Olkin) value. The KMO index is utilized to make a contrast among the enormities of the observed correlation coefficient and partial correlation coefficient (Kaiser, 1974). According to Kaiser (1974), the KMO values should not be <0.5. According to the generally accepted criteria of the statisticians, the variables with Eigenvalues of more than 1.00 are suitable for the analysis. It is evident in Table 8 that all the Eigen values are more than 1.00, which shows that all the variables are fit for analysis. The values of the variance also range from 63.445 to 70.559 and Bartlett's significance values evidently explain that variables are deemed fit for the analysis. Due to the wide usage of SPSS in the studies of social sciences, this software has been applied in this study for analysis purpose. Furthermore, factor analysis has also been carried out in the study. Factor analysis is basically to make the complex and diverse hypothesized relationships simpler. This simplification of the relationships involves unveiling the unrelated variables. Since this study also aims to investigate the complex relationships among the variables, the factor analysis has been conducted using Statistical Package of Social Sciences.

The article "Role of Extrinsic Cues in the Formation of Quality Perceptions" was published in 2022. Journal: Front Psychol.

**Table 8:** Factor analysis.

**Construct**	**No. of items**	**Items**	**Factor loading**	**KMO**	**Barttlet sig**.	**Eigen value**	**% variance**	**Cronbach alpha**
Brand name	5	BN1 BN2 BN3 BN4 BN5	0.545 0.735 0.745 0.716 0.775	0.749	0.00	1.066	70.559	0.836
Country of origin	4	COO1 COO2 COO3 COO4	0.527 0.753 0.740 0.518	0.768	0.00	2.538	63.445	0.806
Price	5	PR1 PR2 PR3 PR4 PR5	0.706 0.562 0.523 0.711 0.653	0.728	0.00	1.089	67.939	0.801
Precautionary label	5	PL1 PL2 PL3 PL4 PL5	0.578 0.683 0.646 0.593 0.769	0.734	0.00	1.042	67.623	0.849
Perceived quality	5	PQ1 PQ2 PQ3 PQ4 PQ5	0.686 0.712 0.757 0.631 0.620 0.650	0.789	0.00	1.485	68.097	0.851
Consumer Knowledge	5	CK1 CK2 CK3 CK4 CK5	0.632 0.574 0.675 0.550	0.800	0.00	5.313	59.032	0.911

### Respondent Profile

For a clear and coherent discussion of results, it is required to comprehend the respondent profile. Table 9 depicts an unambiguous canvas of the respondent profile. The number of respondents used for analysis in the study is 478. The results show that among the total participants of the survey, 59.6% of them were females whereas 40.4% of them were males. High school qualification was possessed by 43.1% of the respondents, and 34.5% among them were bachelors. In total, 24.5% of the respondents acquired a master's degree whereas 7.1% were doctorates. In total, 33.5% of the respondents fall into the age group of 18–25years. In total, 34.9% were within the age group of 26–33years and 24.5% of the consumers were within the age limit of 34–41 years. Only 7.1 of the remaining consumers were 41 years and above.

The article "Role of Extrinsic Cues in the Formation of Quality Perceptions" was published in 2022. Journal: Front Psychol.

**Table 9:** Respondents' profile.

**Demography**	**Indicator**	**Frequency**	**Percentage**
Gender	Male	193	40.4
	Female	285	59.6
Education	High school	206	43.1
	Bachelor	167	34.9
	Masters	71	24.5
	Doctorate	34	7.1
Age group	18–25	160	33.5
	26–33	167	34.9
	34–41	117	24.5
	41-above	34	7.1

### Path Coefficient and Significance Test

This particular study implants structural equation modeling (SEM) for hypothesis testing. Partial least squares (PLS) do not require any assumptions of sample size, normality, etc. Tests for normality such as skewness, kurtosis, and Kolmogorov-Smirnov are not required for using smart PLS. It is free of any kind of limiting constraints which makes it a good choice for data analysis and hypothesis testing. Both approaches factor analysis and path analysis can be used in structural equation modeling. SEM being a unification of both the approaches, concurrently examines both the facets of the model which are the measurement model and structural model.

For testing the hypotheses of the study, the significance level and *t*-values are used (Hair et al., 2011). The path coefficients are standardized beta values. The values of coefficients range from +1 to −1. The strong positive relationship is signified by the values which are closer to +1 and a strong negative relation is depicted by the values which are closer to negative 1 (Henseler et al., 2009). When the signs of the path coefficients are opposite to the hypothesized direction, the hypothesis is not retained. The paths that are empirically supported exhibit the sign which is in line with the hypothesized direction (Hair et al., 2013) (Table 10).

**Table 10:** Path co-efficient and significance level.

**Construct name**	**B-values**	***T*-values**	***P*-values**
Brand name (BN)	0.123	2.873	0.004
Country of origin	0.025	0.622	0.534
Price (PR)	0.081	1.927	0.055
Precautionary label (PL)	0.272	4.512	0.000
BN × CK	0.121	1.698	0.090
COO × CK	−0.130	2.134	0.033
PR × CK	0.054	1.496	0.135
PL × CK	0.054	1.201	0.230

Primarily, the function of the algorithm was applied to produce the path coefficients. Multi-collinearity occurs when two exogenous variables are highly correlated with each other (Hair et al., 2010). According to Chatterjee and Yilmaz (1992), having high multi-collinearity increases the chances of errors and damages the regression values. Although using PLS minimizes the need for normality tests, Hair et al. (2010) suggests the need for a multi-collinearity test prior to examining any theoretical model. Table 11 shows that coefficients of correlations were <0.90, tolerance values were above 0.20, and Variance Inflation Factor (VIF) values were within the range of 1 and 2, which indicate that no issue correlation existed. Thus, multi-collinearity did not exist in the study.

The article "Role of Extrinsic Cues in the Formation of Quality Perceptions" was published in 2022. Journal: Front Psychol.

**Table 11:** Multicollinearity test.

**Variables**	**Tolerance**	**VIF**	**Condition index**
Brand name	0.725	1.380	14.374
Country of origin	0.684	1.462	17.074
Price	0.547	1.828	22.723
Precautionary label	0.422	2.368	26.194
Consumer knowledge	0.976	1.025	32.353

The goodness of fit (GOF) of the model is estimated after the analysis of the predictive relevance of the model. The globally accepted standards for the goodness of fit according to Wetzels et al. (2009) are 0.10 (small), 0.25 (medium), and 0.36 (large).


$$\begin{array}{l} \text{GOF}=\sqrt{\left(\bar{R2}\times \;\bar{AVE}\right)}\\ \text{GOF}=\sqrt{0.478\times \;0.524}\\ \text{GOF}=0.5 \end{array}$$

Furthermore, as a next step, bootstrapping is carried out with a 500 sample size. The sample size selected while running Smart PLS must be greater than the actual sample size which is a condition recommended by Hair et al. (2013). After determining the goodness of fit of the model, path coefficients are determined. The path coefficients are used in order to inspect the hypothesized relationships. The predictable *t*-tests are not assessed in PLS (Barclay et al., 1995). Non-parametric procedures such as bootstrapping are used for the generation of the significance of tests. This study utilized bootstrapping technique which is implanted in Smart PLS to check out the statistical significance of the path coefficients. The variable that interacts with the predictor variable to elucidate the criterion variable is called a moderator variable (Baron and Kenny, 1986). The interaction takes place when the impact of the independent variable on the dependent variable fluctuates with the level of a third variable known as the moderator. In this study, consumer knowledge is used as a moderator for the hypothesized relationships. The interaction latent construct has been established using the product indicator approach. Six interaction effects have been created in this study. The interaction latent constructs of Brand name **×** Consumer knowledge (BN **×** CK), country of origin **×** Consumer knowledge (COO **×** CK), Price **×** Consumer knowledge (PR **×** CK), Precautionary label **×** Consumer knowledge (PL **×** CK) have been examined using bootstrapping procedure with 500 samples. Table 12 exhibits the summary of the regression findings.

The article "Role of Extrinsic Cues in the Formation of Quality Perceptions" was published in 2022. Journal: Front Psychol.

**Table 12:** Path coefficients of hypotheses.

**Hypotheses**	**Relationships**	**B-values**	***T*-values**	***P*-values**	**Decision**	**Impact**
H_1_	BN→PQ	0.123	2.910	0.004	Supported	Major
H_2_	COO→PQ	0.027	0.646	0.519	Rejected	Null
H_3_	PR→PQ	0.082	2.056	0.040	Supported	Minor
H_4_	PL→PQ	0.272	4.620	0.000	Supported	Major
H_5_	BN × CK	0.121	1.698	0.090	Supported	Minor
H_6_	COO × CK	−0.130	2.134	0.033	Supported	Minor
H_7_	PR × CK	0.044	0.814	0.416	Rejected	Null
H_8_	PL × CK	−0.133	1.201	0.230	Rejected	Null

**H**_**1**_**:** The results after hypothesis analysis (β = 0.123, *t* = 2.910, *p* = 0.004) show that H_1_ is supported. It is therefore confirmed that the brand name shows a significant impact on the perceived product quality.
**H**_**2**_**:** The outcomes of the study (β = 0.027, *t* = 0.646, *p* = 0.519) indicate that no significant impact of country of origin on perceived product quality has been noticed which implies that the second hypothesis is rejected.
**H**_**3**_**:** A significant relationship between price and perceived product quality has further been hypothesized. The outcomes (β = 0.082, *t* = 2.056, *p* = 0.040) show that the hypothesis is supported.
**H**_**4**_**:** It was further been hypothesized in the study that precautionary labels cast a significantly positive impact on the perceived product quality and the outcomes confirm that hypothesis has been supported (β = 0.272, *t* = 4.620, *p* = 0.000).
**H**_**5**_**:** As the results reveal that the interaction effect for consumer knowledge among the relationship between brand name and perceived product quality is supported (β = 0.121; *t* = 1.698; *p* = 0.090). The results indicate that high the level of consumer knowledge regarding the brand, the better will be the quality perception of consumers regarding the packaged food product.
**H**_**6**_**:** The hypothesis stated that consumer knowledge moderates the relationship between country of origin and perceived product quality. The bootstrapping results signify that consumer knowledge negatively moderates the relationship between the country of origin and perceived product quality (β = −0.130; *t* = 2.134; *p* = 0.033).
**H**_**7**_**:** The next hypothesis of the study under discussion is that consumer knowledge moderates the relationship between the price and the perceived product quality. However, the outcomes (β = 0.054; *t* = 1.496; *p* = 0.135) reveal that consumer knowledge does not moderate this relationship; hence, the hypothesis is rejected.
**H**_**8**_**:** The moderating impact of consumer knowledge is not confirmed in the relationship between precautionary labels and perceived product quality; hence, the hypothesis that consumer knowledge significantly moderates the relationship between the precautionary label and the perceived product quality is not supported (β = 0.054; *t* = 1.201; *p* = 0.230).

The article "Role of Extrinsic Cues in the Formation of Quality Perceptions" was published in 2022. Journal: Front Psychol.

## Discussion of Findings

The hypotheses of the study have been devised by keeping in view the objectives of the study. The major aim of this study is to find out the impact of extrinsic packaging cues on the quality perceptions of consumers. The brand name is taken as an independent variable and the perceived product quality is taken as a dependent variable. In order to confirm the first hypothesis, PLS bootstrapping technique has been employed. The prevalence of a positive and significant relationship between brand name and perceived product quality can be ascribed to the likelihood that brand name as a packaging element is considered an essential quality cue. The brand name aids the consumer to develop perceptions regarding the packaged food product. The result of the hypothesis could also be explained as product quality is judged by the consumer prior to the usage by taking into consideration the brand name. The outcomes of Qasem et al. (2016) and Zafar et al. (2017) whose findings also reveal that brand name casts a positively significant impact on the quality perceptions of the consumers. It can be inferred from the findings of the study as well as the coherence with the past studies that brand name is an extrinsic cue that is considered by the consumer to predict the quality. Moving on further to the second hypothesis of the study it can be seen that no impact of country of origin prevails on perceived product quality. The absence of a significant relationship between the variables can be attributed to the fact that the impact country of origin cue is subjugated in the presence of other marketing cues. The other cues for instance brand name, price, etc. overpower the effect of the country of origin. The results can further be explained that Pakistani consumers are less aware of the country of origin labeling as most of the research is being carried out in the European markets. Rezvani et al. (2012) and Kalicharan (2014) have also investigated the nexus of the variables and found out that the impact of the country of origin gets dominated by the presence of other variables.

Furthermore, the third hypothesis of the study considers the impact of price on the perceived product quality. The positively significant relationship possibly emerges from the fact that Pakistani packaged food consumer is becoming health-conscious, they expect the value from the product in exchange for money, and they believe in the genuineness of the product. According to the findings of Miyazaki et al. (2005) and Yang et al. (2019), the price of the product is a sheer indicator of quality for the consumers prior to its actual usage which also coincides with the outcomes generated by this particular study. The quality indication ability of the price not only holds true in Pakistan but all around the globe. The subsequent fourth hypothesis proposed an effect of precautionary labels on perceived product quality was successfully supported. The substantial relationship between precautionary labels and perceived product quality arises from the likelihood that international and Pakistani consumers are suffering from various kinds of food allergies tend to have an inclination toward the presence of precautionary labels and contemplate the packaged food with this label of good quality in comparison with the products without any such display of information. The impact of precautionary labels on quality perceptions formed by the consumers regarding the enclosed product has been previously studied by Noimark et al. (2009) and Zurzolo et al. (2013). The results of the study coincide with the outcomes of the findings of the stated scholar in which a significant impact of precautionary labels has been found on quality perceptions.

The article "Role of Extrinsic Cues in the Formation of Quality Perceptions" was published in 2022. Journal: Front Psychol.

Furthermore, it has been hypothesized that the consumer acts as a moderating variable in the framework. The knowledge acquired by the consumers regarding extrinsic cues aids in the formation of product quality perceptions. The fifth hypothesis of the study proposes a significant interaction effect of consumer knowledge on the relationship between the brand name and the perceived product quality is found to be retained. The observed interaction impact of consumer knowledge reveals that with changing levels of consumer knowledge, the consumers' perceived product quality toward the brand name also changes. The impact of consumer knowledge as a moderator has also been tested by Brucks (1985) and Rao and Monroe (1988) who revealed that quality perceptions of the consumers are impacted by the brand name where the consumer knowledge acts as a moderator. The subsequent hypothesis H_6_ proposes that consumer knowledge moderates the relationship between the country of origin and the perceived product quality. The hypothesis is seen to be retained at a minor level by the results. The prevalence of a slight moderating effect shows that with the varying levels of consumer knowledge the quality perceptions of consumers formed through the country of origin label also fluctuates. The relationship however is being supported with a negative sign, which indicates that increased consumer knowledge results in a decreased level of quality perceptions. The results are contrary to the findings of various studies being carried out in European consumer markets. Put differently, the results can be explained that consumers of Pakistan are not well aware of the concept of country of origin so far because of the lack of research as well as the impact of the country of origin label is minimal in the presence of other marketing cues (Kalicharan, 2014).

The article "Role of Extrinsic Cues in the Formation of Quality Perceptions" was published in 2022. Journal: Front Psychol.

The seventh hypothesis asserts that consumer knowledge interacts with the relationship between price and perceived product quality. The results indicated that consumer knowledge shows no moderating effect on the relationship. The fluctuating levels of consumer knowledge regarding the price do not lead to any fluctuations in the levels of perceived product quality. Alternatively, with the high or low levels of knowledge related to pricing, the Pakistani consumer tends to behave correspondingly. The study conducted by Capraro et al. (2003) and Veale and Quester (2009) revealed a very minimal and weak effect of consumer knowledge as a moderator in a similar kind of relationship testing. The final hypothesis declares that the relationship between precautionary labels and perceived product quality is moderated by consumer knowledge is seen not to be retained. Consumers with a high or low level of consumer knowledge tend to behave similarly while forming quality perceptions toward precautionary labels. It has further been confirmed by Choi and Choi (2016) and Soon (2018) also consider that consumer knowledge does not hold as a moderator which confirms the findings of the above study.

## Contributions

### Theoretical Contribution

From a theoretical point of view, this study is significant in the following ways. For instance, this study presents a comprehensive model for understanding the consumer quality perceptions formed based on food packaging cues. A limited number of studies have focused on the Pakistani consumer market. It widens the knowledge base by highlighting the relation between the concept of food packaging and product quality perception. Unlike the developed world, there is minimal research work on food packaging cues in developing countries. Marketing all around the world is changing. The attractive packages are becoming a major tool for communication and perception formation. The packaging of food products is also becoming innovative. The food packages have visual representations which the consumers see and respond to. The consumers of Pakistan are attracted to labeling and are conscious of the quality they perceive from these labels but there is a lack of understanding. This research would contribute to the generalizability of the signaling theory. This research bridges the gap by providing insight into the consumer market of a developing country. The contribution of the study to the literature by testing the existing theory and its generalizability to the Pakistani context is undeniable. However, the significance of the investigation is that it offers comprehensive information about the product quality perceptions formed based on extrinsic food packaging cues.

The article "Role of Extrinsic Cues in the Formation of Quality Perceptions" was published in 2022. Journal: Front Psychol.

### Practical Contribution

Along with theoretical contributions, this study has made few methodological contributions as well. This study uses the mall intercept method as a sampling technique. Nevertheless, this study is a footstep ahead in considering very little detail in terms of gate sampling and day and time sampling. This study also anticipates the upcoming researchers to achieve data from the mall intercept technique. Second, although the reliable items of measures are adopted/adapted from various sources, the studies are conducted in dissimilar situations. In such circumstances, it becomes imperious to establish validity and reliability. This study has comprehensively done various statistical calculations in order to establish the validity and reliability of the Pakistani consumer market. This research now offers a valid and reliable instrument for Pakistani as well as global researchers who are enthusiastic to probe into the product quality perceptions formed *via* food packaging cues.

The consumer trusts the brands which succeed to maintain a high-quality level. In order to maintain the perception of quality, compliance with the regulatory mechanisms is also needed. The lost consumer trust in product quality is quite costly, and it might take forever to regain the public trust. Blockchain technology provides the surety to maintain quality. These un-modifiable records can be referenced much more quickly and accurately than traditional systems, thus helping to guarantee consumer and regulatory confidence.

## Future Directions

In the next future, the supply chain and the blockchain applications will be interested in radical transformation. In this context, a pivotal role concerns the time-limited privacy in blockchain and transactional privacy, enabling applications where privacy is managed and guaranteed by regulations. Furthermore, a research direction concerns the necessity to conduct further research on the role of blockchain technology in managing trust, traceability, and transparency of public and private companies operating in developing countries to underline the research advancements and highlight similarities and differences with developed countries. Finally, an additional research direction concerns the opportunity to adopt blockchain to bridge trust, traceability, and transparency factors affecting knowledge flows during pandemics. To achieve this aim, future contributions could design novel blockchain models to assure the immediate need for personal protective equipment (PPI) such as medical gowns, surgical masks, and gloves, as well as the acquisition and deployment lifecycle of equipment such as ventilators respirators, and medical tests. More in detail, future contributions could provide fertile ground for experimentation of private and permissioned blockchain platforms to manage the material and information flow of PPI supply processes, including different actors, namely medical device suppliers, pharmacies, hospital procurement departments, and local governments.

The article "Role of Extrinsic Cues in the Formation of Quality Perceptions" was published in 2022. Journal: Front Psychol.

## Conclusion

The overall research findings can be concluded as extrinsic cues that possess a significant and positive impact on quality perceptions. The food packaging cue of the brand name showed a positive significance on perceived product quality. Afterward, the country of origin was taken as an extrinsic cue whose result was insignificant. The next extrinsic cue which is tested in the study is price, which exhibited a positive significant relationship with the perceived product quality. Furthermore, the nutritional label was another cue that was employed in the theoretical framework of the study. The extrinsic cue of the nutritional label also significantly impacted perceived product quality. The other two extrinsic cues that were put to analysis were the precautionary label and the Halal logo. Both showed considerable impact on the perceived product quality. Considering the outcomes, the marketers are left with a single choice to take into consideration the packaging and labeling as noticeable extrinsic cues. Consumer knowledge was the intervening variable being employed in the study; the overall impact emerged less strongly. However, consumer knowledge acted as a moderator in the relationships of the country of origin and the brand name with the perceived product quality. As the wave of using packaged food products is recent in Pakistan, hence the impact of knowledge came out to be comparatively weak. The initial framework conceptualized for the study was further strengthened by the signaling theory. The extrinsic cues whose effect on perceived product quality was a matter of interest for the researcher came out to be effective indicators of quality (pre-trial). The findings confirm that the model was in line with the underlying theory. As a concluding remark, a need exists on the edge of marketers of Pakistan to recognize these extrinsic cues in the packaged food product as key drivers for quality perception. Since no study is free of limitations, researchers could not use experimental design due to scarce financial and time resources. Therefore, future researchers can use the experimental design for testing these hypotheses.

The article "Role of Extrinsic Cues in the Formation of Quality Perceptions" was published in 2022. Journal: Front Psychol.

## Data Availability Statement

The raw data supporting the conclusions of this article will be made available by the authors, without undue reservation.

## Ethics Statement

The studies involving human participants were reviewed and approved by University Utara Malaysia. Written informed consent for participation was not required for this study in accordance with the national legislation and the institutional requirements.

## Author Contributions

AJ: manuscript writing and data analysis. ZM: data gathering. ZK: literature review. MA: analysis and interpretation. All authors contributed to the article and approved the submitted version.

## Funding

MA received a fund from the Researcher Supporting Project number (RSP2022R481), King Saud University, Riyadh, Saudi Arabia, to support the publication of this article. The funding agency had no role in designing the study, conducting the analysis, interpreting the data or writing the manuscript.

## Conflict of Interest

The authors declare that the research was conducted in the absence of any commercial or financial relationships that could be construed as a potential conflict of interest.

## Publisher's Note

All claims expressed in this article are solely those of the authors and do not necessarily represent those of their affiliated organizations, or those of the publisher, the editors and the reviewers. Any product that may be evaluated in this article, or claim that may be made by its manufacturer, is not guaranteed or endorsed by the publisher.
